# Clinical Efficacy and Safety of Anterior Cervical Decompression versus Segmental Fusion and Posterior Expansive Canal Plasty in the Treatment of Multilevel Cervical Spondylotic Myelopathy

This article has been retracted.

**DOI:** 10.1155/2022/7696209

**Published:** 2022-04-11

**Authors:** Chen Xia, Fangfang Shi, Chuyong Chen, Jun Lv, Qi Chen

**Affiliations:** ^1^Department of Orthopedics, Zhejiang Provincial People's Hospital, People's Hospital of Hangzhou Medical College, Zhejiang, Hangzhou 310014, China; ^2^Department of Hematology, Zhejiang Provincial People's Hospital, People's Hospital of Hangzhou Medical College, Zhejiang, Hangzhou 310014, China

## Abstract

**Objective:**

To compare the clinical efficacy and safety of anterior cervical decompression and segmental fusion and posterior expansive canal plasty in the treatment of multisegment cervical myelopathy.

**Methods:**

Retrospective analysis was performed of 56 cases of multisegment cervical myelopathy patients admitted from July 2018 to June 2021, 32 male patients and 24 females, aged 56.9 ± 12.8 years with an average duration of 10.6 ± 3.2 years. All patients' preoperative imaging examination revealed multiple-segmented cervical disc herniation and had clinical manifestations of cervical myelopathy.

**Results:**

No neurovascular complications occurred in both groups, and 24 to 36 months of follow-up (mean 28.6 months) were obtained. The height of the cervical spondylosis segment was higher than that 2 weeks after surgery (*p* < 0.05), and the curvature of the cervical spine was significantly lower than that before surgery. There was no statistical significance in the height of the anterior column and curvature of the cervical vertebra at 2 weeks after surgery and at the last follow-up (*p* > 0.05). There were statistically significant differences in anterior curvature of the cervical spine between the two groups at 2 weeks after surgery and the last follow-up (*p* < 0.05). Japanese Orthopaedic Association (JOA) scores in both groups recovered significantly after surgery. At 3 months and the last follow-up, the improvement rate of JOA score in the anterior approach group was significantly higher than that in the posterior approach group (*p* < 0.05), and the improvement rate of JOA score in the anterior approach group was also better than that in the posterior approach group (*p* < 0.05).

**Conclusion:**

This segmented anterior fusion procedure can effectively restore the anterior cervical column height and can significantly improve spinal cord function compared with posterior spinal canal enlargement plasty, thus could be considered an effective option for the treatment of multisegment cervical myelopathy.

## 1. Introduction

Osteophytes at the posterior edge of the vertebral body are a common cause of cervical spondylotic spondylosis, and cervical spondylosis (CS) is caused by multiple segment cervical spine degeneration which is not uncommon in clinical practice [1, 2]. For cervical spondylotic myelopathy (CSM) caused by multiple segment cervical spine degeneration, the compression of the spinal cord or nerve root is generally alleviated by direct anterior decompression or posterior indirect decompression, to achieve the purpose of improving the symptoms [3]. However, for multiple segment disc herniation of patients with CS, after anterior decompression often need to fix multiple cervical segments. Long segment cervical fusion for cervical physiological curvature is very big and is bound to affect the normal biomechanical characteristics of the cervical spine. Moreover, long-segment fusion surgery for the influence of adjacent segment degeneration is still controversial in the world [4–6].

The efficacy of anterior cervical surgery, as one of the main surgical methods of treating CS, has reached a consensus since the procedure was invented in the 1960s [7]. The principle of this operation is to achieve direct decompression through the removal of the posterior margin hyperplasia or the protruding cervical disc [8]. In addition, anterior surgery can open the diseased intervertebral space or vertebral body to restore the vertebral height, and then make the lesion segment fusion through bone grafting, thus eliminating the possibility of the continued lesion in this segment. Such surgery can not only restore the height of CS degeneration, but also restore some or all of the cervical anterior convex physiological curvature, thus holding open the folded yellow ligament, and then expanding the volume of the cervical canal and nerve root canal [9]. However, for the anterior cervical surgery with long segments, especially the anterior cervical surgery fixed with a long titanium cage and anterior long titanium plate, the normal biomechanical state of the cervical spine will be significantly changed. Therefore, it is considered to increase the risk of adjacent segment degeneration after surgery [10]. Although there are pathological changes in multiple plane vertebral body, disc, spinal canal, and spinal cord in long segment CS, there is no consistent understanding of whether they can cause clinical symptoms, whether phase I surgical decompression is needed, or which surgical choice is needed [11].

In this study, 56 patients cases with multilevel cervical spondylotic myelopathy (CSM) from July 2018 to June 2021 who were treated with anterior decompression and segmenting fusion and posterior expansive canal plasty respectively were retrospectively analyzed to evaluate the clinical efficacy and safety of these treatment options.

## 2. Materials and Methods

### 2.1. Basic Clinical Features of Patients

Inclusion criteria for the cases: Those cases that had clinical manifestations of cervical myelopathy, radiographic continuous multisegment cervical disc herniation; no serious cardiovascular and pulmonary diseases, can tolerate surgery, and can cooperate with long-term clinical follow-up were included. There were 56 cases in this group, including 32 males and 24 females. The average age was (56.9 ± 12.8) years. Preoperative CT or MRI examination showed multilevel cervical disc herniation and clinical manifestations of CSM, such as weakness of lower limbs, feeling of stepping on cotton, decreased muscle strength of lower limbs or limbs, increased muscle tension of lower limbs, active or increased antireflex of limbs, positive pathological signs such as Hoffmann's sign and Babinski's sign. Preoperative JOA scores ranged from 4 to 12, with an average of (8.2 ± 0.8) points. Thirty-four patients were treated with segmental anterior cervical interbody fusion device plus titanium cage and titanium plate internal fixation, and 22 patients were treated with posterior C_3_–C_7_ single-door expansion canal plasty. The follow-up period was 24–36 months (Table 1). This is a retrospective study approved by the ethical committee of the Hospital. The informed consent approval was not required as anonymized patient data was used in this study.

### 2.2. Therapeutic Methods

#### 2.2.1. Anterior Group

Anterior cervical discectomy and fusion(ACDF)were performed. For example, the disc herniation of C_3,4_, C_4,5_, C_5,6_ was introduced as an example. After general anesthesia, the supine position was taken and the towel was routinely disinfected. The right transverse incision before the neck was taken, the skin, subcutaneous tissue, and platysma myoides were cut successively, entering the gap between the tracheal and oesophageal sheath and the cervical vascular sheath, exposed to the anterior edge of the vertebral body, and oesophageal; then, a positioning needle was placed. Form X-ray, the gap was confirmed, placed open screws and automatically opened in C_3_, C_4_ vertebrae, open C_3,4_ intervertebral space, C_3,4_ disc full decompression, nerve dissection without obvious nerve compression, appropriate size cage with autologous or allogeneic bone in the C_3,4_, released the moderate pressure, and then in C_4,5_, C_5,6_ intervertebral gap, removed C_4,5_, C_5,6_. The disc was subtotal with parallel C_5_ vertebra, and the appropriate size cage with autologous or allogeneic bone titanium cage was placed. Then a appropriate size plate was inserted and fixed. After the X-line of the C-shaped arm confirmed that the built-in position was in good condition, the wound was fully washed with hydrogen peroxide, normal saline, and olonidazole in turn, and the smoke roll drainage strip was placed, confirming that the device dressing was correctly placed, and then the wound was closed by the layer.

#### 2.2.2. Posterior Group

For posterior C_3_–C_6_ open-door dilated spinal canal plasty, a prone position was taken after general anesthesia, and a conventional disinfection blanket was used. A median incision was taken at the back of the neck, exposing cervical C_3_–C_6_ lamina to bilateral facet joints, grinding 1/2 of the lamina full-thickness bone at the junction of the right lamina and facet joints, grinding full-thickness lamina bone at the junction of the left lamina and facet joints, and release C_2, 3_, The C_6,7_ interlaminar ligament was connected, the left C_3_, C_4,_ C_5_and C_6_ were fixed with small titanium plates between lamina and facet joints. After confirming that the X-line of the C-shaped arm is correct, the wound was fully washed with hydrogen peroxide, normal saline, and olonidzole, and the negative pressure drainage bottle was placed, confirming that the device dressing is correct, and then the wound was closed according to the layer.

The above two groups were followed for 3 months after postoperation, and the drainage strips (or drainage bottles) were removed from 24 to 48 h after surgery. Besides, hormones, antibiotics, and neurotrophils were routinely monitored after surgery. The lower ground activity started from 1 to 2 days after surgery.

### 2.3. Indicators and Methods of Observation Results

At 2 weeks after surgery, different observations at posterior-anterior, lateral, overextended flexion dynamic positions were noted. (1) Clinical observations: During the follow-up period, the subjective symptoms of the patient's subjective symptoms (mainly related to CS, such as the sensation of both limbs, muscle strength, the cotton feeling of stepping in both lower limbs) were observed. (2) Imaging observations: the height of the cervical anterior column by applying the preoperative and postoperative X-ray slices of the cervical spine was noted. The height of the anterior cervical spine column was used to measure the connection between the middle point of the upper edge. The length of the line reflects to be resected and the height of the disc to be removed. The measurement method of anterior cervical curvature was to perform the lower edge of the C_7_ vertebral line and the middle point of the nodules before and after the Atlas and then do two vertical lines respectively, and the upper Angle of the two vertical lines is the anterior curvature Angle of the cervical vertebra. (3) Efficacy evaluations: JOA scores before surgery were recorded and at each follow-up, according to the orthopedic Society of Japan. The postoperative improvement rate was also calculated according to the following formula:

Improvement rate = ((follow-up score preoperative score)/(17-preoperative score)) 100%.

### 2.4. Imaging Observation

The fusion time and fusion rate were observed by imaging and the Cobb angle was measured. Cobb angle calculation was performed as two vertebrae with the anatomical position were selected; a straight line along the upper edge and the lower edge was drawn and made their vertical lines, and the Angle of the intersection of two vertical lines was considered as Cobb angle (Table 2).

### 2.5. Evaluation of Neural Function

The neural function was evaluated according to the JOA scoring standard using the formula below:

Improvement rate = (postoperative score-preoperative score)/(17 - preoperative score) × 100%. The following categories were made according to the results observed.

Excellent: 75%; good: 50%∼74%; middle: 25%∼49%; bad: 24%.

### 2.6. Statistical Analysis

SPSS 23.0 software (IBM USA) was used for statistical analysis of all data of this study. Measurement data (anterior vertebral column height, anterior cervical curvature, JOA score, and improvement rate) are expressed as the mean standard deviation of (*x* ± *s*), using a two-sample mean *t*-test. *p* < 0.05 was considered to be statistically significant.

## 3. Result

### 3.1. Routine Clinical Outcome Index Observation

All patients were followed up for 24–36 months (28.6 months on average). The nervous system (sensory and motor function) of 56 patients was improved to varying degrees after surgery. Most patients had significant improvement in limb mobility, weakness of lower limbs, and feeling of stepping on cotton were significantly reduced, and walking was more stable and powerful than before surgery.

### 3.2. Imaging Observation

No built-in complications such as insert loosening, displacement, sinking, and steel plate fracture were found during the follow-up. The results of the anterior column height and anterior cervical curvature of the two preoperative procedures, 2 weeks after surgery, and at the last follow-up are presented. While the anterior postheight was slightly lost at the last follow-up, it was not statistically significant (*p* > 0.05) (Figure 1).

In the posterior approach group, there was no statistical significance in the height of an anterior column of the lesion segment 2 weeks after surgery and at the last follow-up (*p* > 0.05). There was no statistically significant difference in anterior column height between the two groups before surgery, but there was a statistically significant difference at 2 weeks after surgery and the last follow-up. In the anterior approach group, cervical curvature at 2 weeks after surgery was significantly lower than that before surgery (*p* < 0.05). Statistical difference was observed between anterior cervical curvature at 2 weeks postsurgery and the last follow-up (*p* < 0.05) (Figure 2).

### 3.3. Spinal Cord Function Score and Its Rate of Improvement

In terms of spinal function recovery, significant postoperative recovery was observed compared to surgery. The JOA scores at 3 months and last follow-up were also statistically significant (*p* < 0.05) (Table 3) between the two groups.

According to the subitem results of the JOA score, both the anterior fusion and posterior spinal canal enlargement groups were significantly improved in upper and lower limb movement and sensory function compared with surgery, and bladder function was not significantly different compared with surgery. By comparing the JOA subscores at 3 months after the two different postoperative procedures, the anterior fusion group was statistically significant in both the upper and lower limb motor scores compared with the posterior spinal canal enlargement group, but no difference between the two groups in sensory function and bladder function was observed. The last follow-up result was similar to that obtained 3 months after surgery. Meanwhile, the rate of improvement of JOA scores between the two groups was also statistically significant at 3 months and the last follow-up (*p* < 0.05), and the anterior fusion group was significantly better than the posterior surgery group (Table 4).

### 3.4. General Observation Results

The time of surgery, intraoperative bleeding, and hospitalization of the patients in the observation group was significantly lower than those in the control group (*p* < 0.01) as shown in Table 5.

### 3.5. Comparison of the Preoperative and Postoperative JOA Scores

There was no significant difference in preoperative JOA scores (*p* > 0.05) of the patients as shown in Table 6. The improvement rate in JOA scores at 6 months (63.8 ± 6.6) was significantly higher than the posterior group (57.5 ± 7.1), and the two groups showed statistically significant differences (*p* < 0.05) (Figure 3).

### 3.6. Differences in Imaging Characteristics between ACDF and LMP

Cervical spondylotic myelopathy is caused by prolapse or degeneration of the cervical disc, causing intervertebral osteosis and compressing the spinal cord. With the acceleration of aging and the accelerated pace of life in China, the proportion of CSM patients with multiple segment involvement at medical treatment gradually increased. Except for those with perioperative complications, the X-ray showed no titanium plate and titanium mesh during the follow-up. According to postoperative X-ray follow-up, bone graft fusion was 6 to 11 months, 84.2% (16/19), 9 to 13 months, and 81.8% (27/33) (Figures 4 and 5).

## 4. Discussion

Multisegment cervical spondylotic myelopathy is not uncommon in clinical orthopedics, and its main clinical characteristics are extensive lesion-involved segments and more serious symptoms [12, 13]. With the development of MRI technology, the diagnosis rate of bone and disc herniated spinal diseases has been significantly improved [14–16]. However, there is still widespread international controversy about how to surgically treat multisegmented cervical pulp compression diseases [17]. Both anterior cervical discectomy and fusion and posterior cervical canal angioplasty are surgical methods for cervical myelopathy [18]. Anterior surgery indirectly expands cervical canal volume by directly relieving local compression of nerves and spinal cord and restoring cervical physiological curvature and intervertebral height, while posterior expansive canal plasty indirectly achieves decompression by directly expanding cervical canal volume [19–21]. The purpose of the anterior surgery of cervical spondylosis is to relieve the spinal cord compression, expand the factors of the cervical spine canal capacity, restore normal spinal canal function, and create conditions for the recovery of the cervical spine pulp function [22]. As the gold standard of anterior cervical fusion, iliac trifacial cortical bone graft fusion has been widely used in anterior cervical surgery for various cervical diseases. Front cervical decompression often destroys the stability of the anterior column, whereas, the height of the graft and the maintenance of the early postimplantation stability is the fundamental guarantee for the recovery and correction of the cervical force lines [23]. Therefore, the recovery and maintenance of cervical physiological curvature and vertebral height are increasingly valued by spine surgery and neurosurgeons [24].

Main problems of continuous multiple segments of anterior cervical spine fusion fixation include: (1) multiple segments of cervical spondylosis due to bone hyperplasia, continuous multiple segments of disc degeneration, cervical disc stenosis, cervical physiological curvature disappear or even reverse pathological changes, continuous multisegment fusion fixation is often unable to correct or even aggravate the cervical curvature change; (2) The loss of vertebral height is inevitable. After long segments of bone absorption at the bone grafting interface (or bone intersite interface), the recovered vertebral height of the intervertebral bone graft could be lost; (3) Changes in the physiological curvature can directly affect the effective volume of the spinal canal. In addition, the loss of intervertebral height may also lead to nerve root compression and produce symptoms of nerve root compression; (4) The fusion of long segments due to the long fixed segment, there is a certain degree of micromovement between the bone grafting interface, which could have an obvious impact on the fusion of bone grafting, which can easily lead to fusion failure or false joint formation; (5) A problem in the long segment fixation may result in or accelerate the degeneration of adjacent segment, the adjacent segment degeneration is caused by natural progression, although there are controversial strategies for the problem currently, long segmental fixation will have on adjacent segment larger biomechanics changes, increased intervertebral disc pressure and facet joint stress in adjacent segments.

The ideal procedure for CSM should maintain both a high fusion rate and the cervical curvature [25–27]. The segmented fusion scheme proposed by the author, due to the use of intervertebral bone grafting and vertebral subtotal bone grafting, has an important role in increasing the stability of the bone graft segment and maintaining the physiological curvature of the cervical vertebra and has its main advantages including (1) Segmental bone grafting allows a “normal” vertebral body to be separated, so that the stress transfer between the two bone graft parts can be normal and the stress transfer after fusion can be effectively reduced; (2) When the cervical spine is extended, the anterior steel plate can play a tension band and absorb the tension of the bone-built-in interface. Whereas the cervical anterior flexion, the steel plate plays a supporting role, which can better maintain the height and physiological curvature of the vertebral space, strengthen the stability of the cervical spine, promote fusion, and improve the fusion rate.

## 5. Conclusion

From the JOA score data found in this study, it is evident that in 3 months after surgery, the upper and lower limb movement and sensory function are significantly improved compared with the two preoperative. Improvement in the upper and lower limb motor function and anterior decompression group has significant advantages over the posterior decompression group. In sensory function, there is no obvious difference between the two groups (*p* > 0.05). This may be associated with the reduction of anterior decompression directly beyond the cortical spinal tract compressing the anterior spinal tract [28]. It plays a vital role in restoring spinal cord function [29]. Posterior spondyloplasty, on the other hand, provides indirect decompression through flotation [30–34]. The decompression effect depends on the available buffer space of the posterior approach, and even if the posterior approach has sufficient buffer capacity, if the anterior compressor is too large, the spinal cord will still be compressed [35]. Moreover, if the spinal cord drifts back too much, it will have a certain degree of pulling effect on the nerve root, resulting in some nerve root symptoms such as numbness and pain in the upper arm [36]. To sum up, segmented anterior fusion surgery can effectively improve the symptoms of patients with multisegmented cervical spondylosis, can restore and maintain the cervical anterior column height to a certain extent, and can have a good effect on postoperative functional recovery.

## Figures and Tables

**Figure 1:** Sagittal MRI(T2) performed before anterior cervical decompression and segmental fusion.

**Figure 2:** Sagittal MRI(T2) was performed before posterior cervical expansive canal plasty.

**Figure 3:** Preoperative and postoperative anteroposterior and lateral radiographs.

**Figure 4:** Comparison of preoperative and postoperative MRI and X-ray in anterior cervical decompression and fusion (ACDF) surgery.

**Figure 5:** Comparison of preoperative and postoperative MRI and X-ray in posterior laminoplasty (LMP) surgery.

**Table 1:** Clinical features of multilevel cervical disc herniation.

Subgroup analysis	Cases (*n*)	Gender		Age (Year)	Time of disease	Distribution of surgical segments	
		Male	Female			C_3_–C_6_	C_4_–C_7_
Anterior group	34	24	10	56.7 ± 12.5	10.2 ± 2.7	26	8
Posterior group	22	8	14	59.1 ± 8.2	10.6 ± 3.6	15	7
*t*		0.212		0.425	0.771	0.562	
*p*		0.345		0.765	0.223	0.501	

**Table 2:** Analysis and comparison of imaging characteristics in different periods.

Time	Anterior group (*n* = 34)		Posterior group (*n* = 22)	
	Vertebral column height (mm)	Curvature of the cervical spine	Vertebral column height (mm)	Curvature of the cervical spine
Preoperative	71.2 ± 1.3	23.4 ± 7.8	70.2 ± 5.2	24.3 ± 7.8
2 weeks after surgery	73.4 ± 2.5	19.5 ± 7.8	71.4 ± 3.9	24.6 ± 6.8
Last follow-up	72.1 ± 4.2	21.4 ± 8.2	69.6 ± 3.9	25.3 ± 6.6

**Table 3:** Analysis and comparison of JOA scores in different periods.

Items	Anterior group (*n* = 34)		Posterior group (*n* = 22)	
	Preoperative	3 months after surgery	Preoperative	3 months after surgery
Upper limb function	1.2 ± 0.8	3.2 ± 0.8	1.1 ± 0.7	2.1 ± 0.8
Lower limb function	1.1 ± 0.8	3.0 ± 0.7	1.1 ± 0.7	2.1 ± 0.8
Sensory function	3.1 ± 0.2	5.1 ± 0.5	3.2 ± 0.3	5.2 ± 0.7
Bladder function	2.2 ± 0.6	2.1 ± 0.7	2.1 ± 0.8	2.1 ± 0.4
Total	8.4 ± 0.8	15.4 ± 0.8	8.2 ± 0.9	13.5 ± 0.2

**Table 4:** Comparison of JOA score before and after the operation.

Subgroup analysis	Case (*n*)	Preoperative	3 months after surgery	6 months after surgery
Anterior group	34	8.25 ± 0.75	16.25 ± 0.75	14.65 ± 0.46
Posterior group	22	8.25 ± 0.88	13.55 ± 0.38	12.46 ± 0.55
*t*		0.852	12.215	9.045
*p*		0.082	0.001	0.001

**Table 5:** Bone graft fusion and Cobb Angle fusion before and after the operation.

Subgroup analysis	Case (*n*)	Osteograft fusion		Fusion segment cobb angle	
		Bone fusion time	Bone fusion rate	Preoperative	3 months after the surgery
Anterior group	34	6.25 ± 1.37	40 (71.43%)	1.55 ± 0.35	8.55 ± 0.56
Posterior group	22	7.65 ± 1.87	16 (28.57%)	1.65 ± 0.22	7.82 ± 0.35
*t*		4.655	0.215	5.262	2.455
*p*		0.001	0.065	0.001	0.002

**Table 6:** JOA score improvement rate.

Time	Anterior group (*n* = 34)	Posterior group (*n* = 22)
Preoperative	79.4 ± 8.7	60.4 ± 7.8
6 months after the surgery	63.8 ± 6.6	57.5 ± 7.1
*t*	9.426	3.004
*p*	0.021	0.042

## Data Availability

The labeled datasets used to support the findings of this study are available from the corresponding author upon request.
